# Study of the G Protein Nucleolar 2 Value in Liver Hepatocellular Carcinoma Treatment and Prognosis

**DOI:** 10.1155/2021/4873678

**Published:** 2021-07-19

**Authors:** Yiwei Dong, Qianqian Cai, Lisheng Fu, Haojie Liu, Mingzhe Ma, Xingzhong Wu

**Affiliations:** ^1^Department of Biochemistry and Molecular Biology, School of Basic Medical Sciences, Fudan University, Key Lab of Glycoconjugate Research, Ministry of Public Health, Shanghai 200032, China; ^2^Shanghai Key Laboratory of Molecular Imaging, Shanghai University of Medicine and Health Sciences, Shanghai 201318, China; ^3^Department of Gastric Surgery, Fudan University Shanghai Cancer Center, Shanghai 200025, China

## Abstract

LIHC (liver hepatocellular carcinoma) mostly occurs in patients with chronic liver disease. It is primarily induced by a vicious cycle of liver injury, inflammation, and regeneration that usually last for decades. The G protein nucleolar 2 (GNL2), as a protein-encoding gene, is also known as NGP1, Nog2, Nug2, Ngp-1, and HUMAUANTIG. Few reports are shown towards the specific biological function of GNL2. Meanwhile, it is still unclear whether it is related to the pathogenesis of carcinoma up to date. Here, our study attempts to validate the role and function of GNL2 in LIHC via multiple databases and functional assays. After analysis of gene expression profile from The Cancer Genome Atlas (TCGA) database, GNL2 was largely heightened in LIHC, and its overexpression displayed a close relationship with different stages and poor prognosis of carcinoma. After enrichment analysis, the data revealed that the genes coexpressed with GNL2 probably participated in ribosome biosynthesis which was essential for unrestricted growth of carcinoma. Cell functional assays presented that GNL2 knockdown by siRNA in LIHC cells MHCC97-H and SMCC-7721 greatly reduced cell proliferation, migration, and invasion ability. All in all, these findings capitulated that GNL2 could be a promising treatment target and prognosis biomarker for LIHC.

## 1. Background

Liver cancer is composed of primary carcinoma and metastatic carcinoma [1, 2]. As far as the most common inducers of carcinoma-associated mortality in the world, primary liver carcinoma ranks second, thus becoming a great public health challenge [3–5]. Primary liver carcinoma consists of liver hepatocellular carcinoma (LIHC), intrahepatic cholangiocarcinoma (iCCA), and other rarely seen neoplasms [6, 7]. Mostly, LIHC occurs in patients with chronic liver disease, and it is generally caused by a vicious cycle of liver damage, inflammation, and regeneration that usually span several decades [8–11]. Like other malignant neoplasms, the widely generated biological alteration in LIHC pathogenesis comprises activated oncogene and inactivated neoplasm inhibitor genes [12]. Since its discovery over 60 years ago, alpha-fetoprotein (AFP) has been the most commonly used biomarker in LIHC management [4, 13, 14]. However, LIHC is classified as a complicated disease accompanied by several risk factors caused pathogenic mechanisms. Thus, to characterize LIHC only by a single biomarker is not feasible. To explore the pathogenesis of LIHC and uncover the candidate biomarkers become urgently needed.

As a protein-encoding gene, the G protein nucleolar 2 (GNL2) is also named by nucleostemin (NS), which is essential for stem cell growth and development [15, 16]. GNL2 is highly expressed in tissues, such as testis and bone marrow [17, 18]. Presently, there are no researches on the particular biological function of GNL2, and little is known about its relationship with carcinoma pathogenesis.

Here, our study is aimed at investigating whether there is an association of GNL2 expression with the prognosis in LIHC patients. In addition, our study also wants to validate its inhibitory effect on LIHC cell proliferation, migration, and invasion by *in vitro* experiments.

## 2. Material and Methods

### 2.1. Identification of the Differentially Expressed Genes (DEGs) in TCGA Database

The Cancer Genome Atlas (TCGA) database, as the National Cancer Institute (NCI) and the National Human Genome Institute (NHGRI) supported the project, was employed to obtain mRNA expression profile of liver carcinoma and normal samples. It could offer all-inclusive maps of the main alterations of genomic in multiple sorts of carcinomas. ∣log_2_ fold change (FC) | >1 and *P* value <0.05 were considered to be parameters for identifying the DEGs. The protein-protein network (PPI) of the selected DEGs was constructed by the Search Tool for the Retrieval of Interacting Genes (STRING) database.

### 2.2. Gene Expression Profiling Interactive Analysis (GEPIA) Database

GEPIA is an interacting online server for the analysis of RNA sequencing data of tumorous and healthy samples from the Genotype-Tissue Expression (GTEx) and TCGA datasets. The URL of GEPIA is http://gepia.cancer-pku.cn. In this study, we used GEPIA to determine GNL2 expression in different stages of liver carcinoma and then perform patient survival analysis and identify similar genes.

### 2.3. Kaplan-Meier Plotter Database

The Kaplan-Meier plotter (https://kmplot.com/analysis/), functioning as a web tool, is used to validate survival biomarkers in the light of meta-analysis. The information of gene expression profile and various survival data comprising overall survival (OS), relapse-free survival (RFS), and disease-specific survival (DSS) come from the well-known public databases, including GEO (only Affymetrix microarrays), EGA, and TCGA. Kaplan-Meier plotter was taken to generate the survival curves of GNL2, and log rank *P* values, as well as hazard ratio (HR) with 95% confidence intervals, were calculated.

### 2.4. Biological Process and Pathway Enrichment Analysis

The top 1000 genes coexpressed with GNL2 (sorted by Pearson correlation coefficient) in LICH-tumor and LICH-normal dataset were identified by GEPIA. To assess the gene-annotation enrichment, we utilized the online tool Enrichr (https://maayanlab.cloud/Enrichr/). Enrichment annotations were presented as Kyoto Encyclopedia of Genes and Genomes (KEGG) pathway and Gene Ontology (GO) biological process. Data were plotted and visualized using an online platform http://www.bioinformatics.com.cn.

### 2.5. Cell Culture and Transfection

The human LIHC cell lines MHCC97-H and SMCC-7721 were obtained from the China Center for Type Culture Collection in 2020 and authenticated by short tandem repeat analysis. All cells were routinely cultured in DMEM medium (Thermo Fisher Scientific, Inc., USA) supplemented with 10% FBS (Thermo Fisher Scientific, Inc., USA) in an incubator with 5% CO_2_ at 37°C. SiRNA targeting GNL2 (si-GNL2) and a negative control siRNA (si-NC) were acquired from GeneCopoeia, Inc. (USA). When MHCC97-H and SMCC-7721 cells confluence reached up to 80% on the following day, they were transfected with indicated siRNAs utilizing Lipofectamine 2000 (Invitrogen, USA) as the manual described. Reduced efficiency of GNL2 was determined by qRT-PCR at 48 h posttransfection. The siRNAs used were as follows: si-GNL2-1, 5′-CACGTGTGATTAAGCAGTCATCATT-3′; si-GNL2-2, 5′-CCATACAAAGTTGTCATGAAGCAAA-3′; si-NC, 5′-UUCUCCGAACGUGUCACGUTT-3′.

### 2.6. Quantitative Reverse-Transcription PCR (qRT-PCR) Assay

Overall RNA was harvested from indicated cells utilizing TRIzol reagent (Invitrogen, USA). qRT-PCR was carried out on a Bio-Rad Single Color Real-Time PCR system (Bio-Rad Laboratories, Inc., USA) with SYBR-Green Real-Time PCR Master Mix (Toyobo Life Science, Japan). *β*-Actin was used as an internal control.

### 2.7. Cell Proliferation Assay

2,000 of si-NC- and si-GNL2-transfected cells were plated in per well of 96-well plates, followed by maintaining 0, 24, 48, and 72 h at 37°C. 10 *μ*l of CCK-8 reagent was added into each well at the indicated time, followed by another 2 h incubation. The wavelength at 450 nm was read in a Varioskan Flash spectrophotometer (Thermo Fisher Scientific, Inc., USA).

### 2.8. Transwell Assay

For cell migration assay, Matrigel needed not to be precoated in the Transwell chamber (Corning, NY). The Transwell upper chamber was added 50,000 si-NC- or si-GNL2-transfected cells suspended in serum-free DMEM medium, and the lower chamber was added DMEM medium with 10% FBS, followed by maintaining 24 h at 37°C. Then, migrated cells underside were rinsed by PBS, fixed by methanol, and stained by DAPI. Positive cells were photographed and counted under a microscope. Five random fields were selected and counted the average. For cell invasion assay, 2 mg/mL Matrigel was precoated in the upper chamber. The remaining procedures were the same as the cell migration assay.

### 2.9. Statistical Analysis

Our data were analyzed by the SPSS software (IBM Corp., USA) and were represented as the mean ± SD. The Student *t*-test was employed to analyze the difference in mRNA expression from TCGA database. The correlation existing in expression and pathological stage of carcinoma was assessed by one-way ANOVA. The differences in survival ratio between highly expressed GNL2 and lowly expressed GNL2 groups were detected by Kaplan-Meier analysis and log-rank test. The Student *t*-test was employed to compare the difference of the si-GNL2-transfected group with the si-NC-transfected group. The great statistical difference indicated *P* < 0.05.

## 3. Results

### 3.1. Identification of the DEGs and Overexpressed Gene GNL2 in LIHC

As indicated before, to define the DEGs in liver carcinoma and normal samples, we obtained gene expression information from TCGA database. Totally, 361 DEGs were selected, comprising 283 genes with increased expression and 78 genes with decreasing expression (Figure 1 volcano plot).  Figure 2 displayed the PPI network, 110 nodes (proteins) and 159 edges (proteins interactions). Besides, it was observed that the degree of GNL2 was high which partly revealed the potential role of GNL2 as a candidate biomarker for LIHC.

### 3.2. Validation of the Relationship between the Stages of Liver Carcinoma and the Expression of GNL2

TCGA database analysis showed that LIHC tumor tissues highly expressed GNL2 in comparison with normal tissues (Figure 3(a)). Then, GEPIA analysis discovered the associations between various pathological carcinoma stages of LIHC patients and GNL2 expression level. It was found that GNL2 expression was significantly associated with the pathological carcinoma stages of LIHC (Figure 3(b), *P* = 0.00163). Our results demonstrated that GNL2 exhibited an important part in clinical practice.

### 3.3. Prognostic Value of GNL2 for LIHC Patients

Subsequently, we employed GEPIA to investigate the relationship of GNL2 expression with LIHC patient's prognosis. Figures 4(a) and 4(b) demonstrated the OS and DFS curves of LIHC patients with different GNL2 expression levels. Kaplan-Meier analysis plus the log-rank test was taken to assess the impacts of the expression of GNL2 on OS and DFS. Compared to the lowly expressed GNL2 group, the highly expressed GNL2 group exhibited a shorter OS and DFS (log rank *P* = 9.2*e* − 06 and 0.011, respectively). Additionally, we further verified that high expression of GNL2 led to poor prognosis in LIHC patients by Kaplan-Meier plotter database analysis. Figures 5(a), 5(d), and 5(g) showed that LIHC patients with highly expressed GNL2 had shorter OS, RFS, and DSS compared to those with the lowly expressed group, in line with the GEPIA analysis. Given the high incidence of hepatocellular carcinoma was mainly due to the prevalence of hepatitis virus infection, we further evaluated the prognosis of LIHC patients stratified according to hepatitis virus infection. The results showed that the hepatitis virus did not affect the prognosis of GNL2 (Figures 5(b), 5(c), 5(e), 5(f), 5(h), and 5(i)).

### 3.4. Biological Process and Pathway Enrichment Analysis

We conducted KEGG and GO enrichment analyses of genes coexpressed with GNL2 in LIHC tumor and normal tissues to validate the function of GNL2 in liver carcinoma.  Figure 6(a) displayed the results of KEGG pathway enrichment, including cell cycle, mRNA surveillance pathway, proteasome, ribosome, RNA transport, DNA replication, Fanconi anemia pathway, ribosome biogenesis in eukaryotes, spliceosome, and homologous recombination.  Figure 6(b) showed the enriched biological processes of the genes coexpressed with GNL2 as the following: rRNA processing (GO:0006364), rRNA metabolic process (GO:0016072), ribosome biogenesis (GO:0042254), mRNA processing (GO:0006397), translation (GO:0006412), RNA splicing via transesterification reactions with bulged adenosine as nucleophile (GO:0000377), mRNA splicing via spliceosome (GO:0000398), gene expression (GO:0010467), cellular macromolecule biosynthetic process (GO:0034645), and ncRNA processing (GO:0034470).

### 3.5. Cell Functional Results of GNL2 Downregulation in LIHC Cells

We transfected siRNAs into MHCC97-H and SMCC-7721 cells to evaluate the effects of ablated GNL2 on cell function (Figures 7(a) and 7(b)). CCK-8 assay data showed that si-GNL2-transfected cell proliferation was significantly hindered in comparison with control si-NC-transfected cells after 24, 48, and 72 h treatment (Figures 7(c) and 7(d)). In addition, Transwell assay data revealed that transfection of si-GNL2 in LIHC cells could suppress invasion and migration abilities (Figures 8(a)–8(d)). Therefore, GNL2 knockdown largely curbed MHCC97-H and SMCC-7721 cell proliferation, invasion, and migration.

## 4. Discussion

LIHC is a malignant neoplasm that often occurs in the liver, which is related to drinking, viral hepatitis, eating moldy food, genetics, etc. [19]. Currently, the studies about LIHC are few. As for LIHC treatment, Kim et al. summarized and discussed clinical researches towards systematical chemical therapy for advanced cancer [20]. Zhang and Zhang found FoxP4 functioned as a tumor promoter in LIHC cells by transcriptionally regulating Slug and highlighted the potential effects of FoxP4 on the prognosis and treatment of LIHC [21]. The early stage is often asymptomatic, and obvious symptoms like liver area pain, fever, and fatigue usually appear in the advanced stage [22]. It is possible to cure LIHC in its early stage, but the treatment is complicated in the middle and advanced stages [23, 24]. Therefore, it is necessary to have a better understanding of the molecular mechanism involved in liver carcinoma initiation and to screen novel biomarkers. In this study, we screened 361 DEGs and GNL2 was one of the significantly upregulated genes. Besides, GNL2 was observed to have a high degree in the PPI network. Thus, we considered GNL2 as candidate biomarkers for LIHC.

NS or GNL3 (nucleostemin) and GNL3-like (GNL3L) are two members of the GNL2 family [25]. The two both comprise an MMR_HSR1 domain, depicted by five GTP binding motifs formed as a cyclic order. The two have a common Grnlp homologous sequence in yeast, highly similar to the sequence in vertebrates. GNL3L is the vertebrate aileron of NS, while GNL2 is single both in vertebrates and invertebrates. NS is a protein playing essentially in stem cell growth and maintenance [15]. However, few pieces of research are conducted to explore the relation between GNL2 and disease. Herein, our study plans to explore the role and function of GNL2 in LIHC.

As far as gene expression information from the TCGA database, GNL2 was highly expressed in LIHC tumor samples compared to that in normal samples, implying GNL2 was a possible oncogene in LIHC. After analysis of the associations between various pathological carcinoma stages of LIHC patients and GNL2 expression, the data revealed that high expression of GNL2 was significantly associated with advanced cancer stages. Kaplan-Meier analysis based on GEPIA and Kaplan-Meier plotter datasets consistently verified that LIHC patients with highly expressed GNL2 exhibited a shorter survival ratio. What was more, *in vitro* knockdown functional experiments demonstrated that reducing GNL2 by siRNA impeded LIHC cell proliferation, migration, and invasion abilities. Based on the above findings, GNL2 was probably considered as a treatment target and a biomarker for LIHC patients' prognosis.

The alteration of ribosome biogenesis often occurs in carcinoma cells due to the rising need for protein synthesis in unrestricted cancer growth [26]. Ribosome biosynthesis is a complicated biological process required for the coordination of multiple factors and a huge cellular energy investment. The ribosome is essential for protein production and therefore is essential for cell survival, growth, and proliferation. Ribosomal biogenesis begins in the nucleolus, including ribosomal RNA synthesis and processing, ribosomal protein assembly, and transport to the cytoplasm [27]. Interference in ribosome biogenesis can promote cell cycle arrest, apoptosis, or senescence and thus is usually associated with carcinoma, aging, and some other related degenerative diseases [28]. The hyperactivation of ribosome biogenesis usually occurs in tumor cells to cope with a rising need in protein synthesis and maintain unrestricted growth [29]. Importantly, the hyperactivation of ribosome biogenesis can be initiated by overexpressing oncogenes or eliminating neoplasm suppressing genes. In our study, we found that GNL2 was largely associated with altered ribosome biogenesis in cancer cells through KEGG and GO enrichment analyses, thereby playing a vital role in carcinoma initiation and progression.

This study has some limitations. First, we did not construct an overexpression vector of GNL2, and we further explored the regulation of GNL2 overexpression on the proliferation, invasion, and migration of LIIHC cells. Secondly, we have not used clinical samples to analyze GNL2 mRNA and protein levels. In future studies, we will collect more clinical samples for analysis of GNL2 mRNA and protein levels.

## 5. Conclusion

To our knowledge, this study reported the function of GNL2 in LIHC for the first time, and the results showed that GNL2 was a new biomarker for predicting the prognosis of LIHC patients. Bioinformatics analysis showed that GNL2 was greatly raised in LIHC, and its overexpression was closely related to cancer stage and poor prognosis. Enrichment analysis suggested that GNL2 was largely related to ribosome biosynthesis which was essential for cancer unrestricted growth. Ablating GNL2 resulted in the reduction of cell proliferation, migration, and invasion abilities. These findings demonstrated that GNL2 could be a promising treatment target for LIHC.

## Figures and Tables

**Figure 1:** Volcano plot illustrated the DEGs existing in liver carcinoma samples and normal ones based on TCGA dataset. Genes with upregulation were presented as the red dot, while those with downregulation were shown as the blue dot.

**Figure 2:** PPI network of the DEGs. Nodes displayed proteins, and edges exhibited the interactions between proteins.

**Figure 3:** Highly expressed GNL2 was in LIHC, and its higher expression was associated with carcinoma stages. (a) To analyze GNL2 expression level in normal and tumor tissues of the liver based on TCGA dataset. ^∗∗∗^*P* < 0.001. (b) Analysis of GNL2 expression level in different liver carcinoma stages based on GEPIA dataset.

**Figure 4:** GNL2 high expression was a poor prognosis factor for LIHC. (a) GEPIA analysis of the OS curves of LIHC patients with highly expressed or lowly expressed GNL2. (b) GEPIA analysis of the DFS curves of LIHC patients with highly expressed or lowly expressed GNL2.

**Figure 5:** Prognosis value of GNL2 in LIHC was confirmed by the Kaplan-Meier plotter dataset. The impacts of GNL2 expression levels on the (a) OS, (d) RFS, and (g) DSS of LIHC patients. The impacts of GNL2 expression levels on the (b) OS, (e) RFS, and (h) DSS of LIHC patients without hepatitis virus infection. The impacts of GNL2 expression levels on the (c) OS, (f) RFS, and (i) DSS of LIHC patients with hepatitis virus infection.

**Figure 6:** KEGG and GO analyses of genes coexpressed with GNL2 in LIHC. (a) Dot bubble chart of enriched GO biological process terms. (b) Dot bubble chart of enriched KEGG pathways.

**Figure 7:** Evaluation of cell proliferation in si-GNL2-transfected LIHC cells. GNL2 expression was reduced in (a) MHCC97-H and (b) SMCC-7721 by si-GNL2. ^∗^*P* < 0.05; ^∗∗^*P* < 0.01. Detection of cell proliferation ability in si-GNL2-transfected (c) MHCC97-H and (d) SMCC-7721 cells by CCK-8 assay. ^∗^*P* < 0.05.

**Figure 8:** Cell functional results of GNL2 downregulation in LIHC cells. Validation of cell invasion capability in si-GNL2-transfected (a) MHCC97-H and (b) SMCC-7721 cells by Transwell assay. ^∗^*P* < 0.05; ^∗∗^*P* < 0.01. Validation of cell migration capability in si-GNL2-transfected (c) MHCC97-H and (d) SMCC-7721 cells by Transwell assay. ^∗^*P* < 0.05; ^∗∗^*P* < 0.01.

## Data Availability

The datasets used and/or analyzed during the current study are available from the corresponding author on reasonable request.
